# Analysis of *Mycobacterium tuberculosis*-Specific CD8 T-Cells in Patients with Active Tuberculosis and in Individuals with Latent Infection

This article has been retracted.

**DOI:** 10.1371/journal.pone.0005528

**Published:** 2009-05-13

**Authors:** Nadia Caccamo, Giuliana Guggino, Serena Meraviglia, Giuseppe Gelsomino, Paola Di Carlo, Lucina Titone, Marialuisa Bocchino, Domenico Galati, Alessandro Matarese, Jan Nouta, Michel R. Klein, Alfredo Salerno, Alessandro Sanduzzi, Francesco Dieli, Tom H. M. Ottenhoff

**Affiliations:** 1 Dipartimento di Biopatologia e Metodologie Biomediche, Università di Palermo, Palermo, Italy; 2 Dipartimento di Medicina Clinica e delle Patologie Emergenti, Università di Palermo, Palermo, Italy; 3 TB Infection Screening Unit, Department of Clinical and Experimental Medicine, University of Naples “Federico II”, Monaldi Hospital, Naples, Italy; 4 Department of Immunohematology & Blood Transfusion and Department of Infectious Diseases, Leiden University Medical Center, Leiden, The Netherlands; 5 National Institute of Public Health and the Environment, Bilthoven, The Netherlands; McGill University, Canada

## Abstract

CD8 T-cells contribute to control of *Mycobacterium tuberculosis* infection, but little is known about the quality of the CD8 T-cell response in subjects with latent infection and in patients with active tuberculosis disease. CD8 T-cells recognizing epitopes from 6 different proteins of *Mycobacterium tuberculosis* were detected by tetramer staining. Intracellular cytokines staining for specific production of IFN-γ and IL-2 was performed, complemented by phenotyping of memory markers on antigen-specific CD8 T-cells. The *ex-vivo* frequencies of tetramer-specific CD8 T-cells in tuberculous patients before therapy were lower than in subjects with latent infection, but increased at four months after therapy to comparable percentages detected in subjects with latent infection. The majority of CD8 T-cells from subjects with latent infection expressed a terminally-differentiated phenotype (CD45RA^+^CCR7^−^). In contrast, tuberculous patients had only 35% of antigen-specific CD8 T-cells expressing this phenotype, while containing higher proportions of cells with an effector memory- and a central memory-like phenotype, and which did not change significantly after therapy. CD8 T-cells from subjects with latent infection showed a codominance of IL-2^+^/IFN-γ^+^ and IL-2^−^/IFN-γ^+^ T-cell populations; interestingly, only the IL-2^+^/IFN-γ^+^ population was reduced or absent in tuberculous patients, highly suggestive of a restricted functional profile of *Mycobacterium tuberculosis*-specific CD8 T-cells during active disease. These results suggest distinct *Mycobacterium tuberculosis* specific CD8 T-cell phenotypic and functional signatures between subjects which control infection (subjects with latent infection) and those who do not (patients with active disease).

## Introduction

Globally, Tuberculosis (TB) accounts for approximately nine million new cases of disease and around two million deaths every year [1]. TB is presenting new challenges as a global health problem, especially with new threats of HIV coinfection and multidrug-resistant and extensively drug-resistant strains of *Mycobacterium tuberculosis* (Mtb). TB is transmitted directly from human to human and the control of the infection depends on early identification and proper treatment of individuals with active disease. However, the lack of accurate diagnostic techniques has contributed to the emergence of TB as a threat to global health. To date, there is no simple, rapid, sensitive and specific test that can differentiate active TB from latent infection, and slowly progressive TB.

T-cells, T-cell derived cytokines and cytotoxic molecules are crucial for protection against TB. Although a role for CD4 T-cells in protection against Mtb is well documented, there is also a large body of evidence derived from human and non human models that suggests an involvement of CD8 T-cells [2]–[5]. CD8 T-cells contribute to control of Mtb infection by mediating specific effector functions, including IFN-γ and TNF-α production upon recognition of mycobacterial antigens [6]–[8], lysis of infected host cells [6]–[9], and direct killing of mycobacteria [5], [10], [11]. A limited number of studies focused on the T-cell repertoire in Mtb infection, demonstrating clonal T-cell expansion in granulomas from subjects with LTBI [12] and changes in the peripheral blood and pleural fluid T-cell repertoire from TB patients [13]. Furthermore, CD8 T-cells specific for numerous mycobacterial antigens can be isolated at high frequency from human and mouse models, consistent with the hypothesis that CD8 T lymphocytes are constantly being stimulated with antigen [9], [10].

However, there are few studies which have compared the frequency, phenotype and function of antigen-specific CD8 T-cells in TB patients and subjects with latent infection (LTBI). Among them, we ourselves previously found that the frequency of Ag85A peptide-specific CD8 T-cells was reduced in tuberculous children before therapy, but increased after therapy to levels similar to those detected in healthy tuberculin skin test positive children. Ag85A epitope-specific CD8 T-cells during active TB were mainly present among central memory cells and produced low levels of IFN-γ and perforin, which recovered after therapy [14]. In a parallel study, Kaufmann and colleagues found clonal expansion of effector-memory CD8 T-cells in older children with TB, with potential impact on course and severity of disease [15]. However, the CD8 repertoire of children could well be different from that in adult individuals given the different clinical manifestation of TB in children and adults; moreover, little is known about the size, quality and specificity of Mtb-specific CD8 T-cell responses in adult patients with active TB disease compared to treated TB and subjects with LTBI.

To start addressing these issues, we have in this study determined the *ex-vivo* frequencies, phenotype and functional properties of HLA-A*0201 CD8 T-cells specific for different peptides of Mtb proteins in adult subjects with LTBI and adult TB patients with active disease, both before and following four months of anti-mycobacterial therapy.

## Results

### *Ex vivo* analysis of circulating epitope-specific CD8 T-cells

To determine the *ex vivo* frequency of peptide-specific CD8 T-cells, PBMC from HLA-A*0201 patients with active TB before (T0) and after four months of chemotherapy (T4) and individuals with LTBI were stained with HLA-A*0201/tetramers and anti-CD8 antibody and analysed by FACS.

Four out of the six selected epitopes (Ag85B p5–13, Esat-6 p82–90, Hsp65 p362–370 and 16 kDa p120–128) were previously identified as CD8 T cell epitopes, while Rv1490 p325–333 and Rv1614 p197–205 are newly identified in this study as candidate epitopes, based upon whole Mtb genome screening for 9-mer peptides sequences with high/intermediate HLA-A*0201 binding affinity (see also Table 1). Moreover, a minimum of three and a maximum of all six tetramers marked the CD8 T-cell response in each group of individuals (data not shown). In all instancies, specificity of tetramer staining was confirmed by the negative data obtained both using tetramer of an irrelevant specificity (the HLA-A*0201/HIV-1 gag peptide p76–84) and staining PBMC from normal, uninfected donors with Mtb tetramers (see Table 2).

**Table 1:** HLA-A*0201 binding of predicted HLA-A*0201 binders.

Peptide		AA sequence	rel IC50
**Rv1490**	p325–333	FLLGLLFFV	2,50
**Rv1614**	p197–205	FLYELIWNV	1,79
**Ag85B**	p5–13	GLPVEYLQV	7
**Esat-6**	p82–90	AMASTEGNV	1,25
**Hsp65**	p362–370	KLQERLAKL	0,25
**16 kDa**	p120–128	GILTVSVAV	2,25
**HBV**	core p47–56	FLPSDYFPSV	1

Peptides were tested for their ability to compete binding of 1.6 µM biotinylated peptide HBV core p47–56 to HLA-A*0201 molecules. The concentration of peptide yielding 50% inhibition (IC50) was deduced from the dose-response curve. One of the six peptides bound to HLA-A*0201 with high affinity (IC50<1 µM), while the other peptides bound the HLA-A*0201 with intermediate affinity (IC50 1–10 µM). Each peptide was tested in at least two separate experiments. Data are expressed as relative (rel) IC50, compared to the IC50 of the standard peptide HBV core p47–56, which was considered as 1.

Values are the mean of rel IC50 of two independent experiments with SE being always <10%.

**Table 2:** *Ex vivo* analysis of frequency of peptide-specific CD8 T-cells.

Tetramer	LTBI	T0	T4	PPD^−^ Healthy Donor
**16 kDa**	0.3	0.13^a^	0.22^c^	<0.01
	(0.19–0.55)	(0.05–0.34)	(0.20–0.72)	
**Rv1490**	0.54	0.19^a^	0.3^c^	<0.01
	(0.16–0.80)	(0.11–0.65)	(0.22–0.36)	
**Rv1614**	0.65	0.30^b^	0.3	<0.01
	(0.58–0.85)	(0.11–0.59)	(0.29–0.45)	
**Ag85B**	0.8	0.60	0.64	<0.01
	(0.56–0.94)	(0.31–0.92)	(0.24–1.35)	
**Esat-6**	0.56	0.29^b^	0.58^d^	<0.01
	(0.33–0.96)	(0.17–0.66)	(0.18–0.92)	
**Hsp65**	0.57	0.41^b^	0.34	<0.01
	(0.42–0.80)	(0.31–0.74)	(0.22–0.58)	
**HIV-1 gag**	<0.01	<0.01	<0.01	<0.01

Cumulative data on the frequencies of the tetramer-specific CD8 T-cells in peripheral blood of subjects with LTBI, patients with active TB before (T0) and four months after therapy (T4). Data are presented as median values while interquartile range is shown in brackets.

^a^ *p*<0.01 and ^b^ *p*<0.05 when compared to values in LTBI subjects.

^c^ *p*<0.05 and ^d^ *p*<0.02 when compared to values in TB patients before therapy (T0).

Although there was considerable variability in the proportions of CD8 T-cells that bound to single tetramers, an immunodominance hierarchy in epitope-specific CD8 T-cell response was found both in LTBI subjects and in TB patients at T0 and T4 (Figure 1A and Table 2). In LTBI subjects, the mean *ex-vivo* frequency of peptide-specific CD8^+^ tetramer^+^ T-cells was 0.8% for Ag85B, 0.66% for Hsp65, 0.65% Rv1614, 0.57% for Esat-6, 0.49% for Rv1490 and 0.43% for 16 kDa. The *ex-vivo* frequency of tetramer-specific CD8 T-cells was higher in LTBI subjects than in TB patients (Table 2) and this difference attained statistical significance with most of the studied epitopes (i.e, Esat-6, Rv1614, Rv1490, Hsp65 and 16 kDa). Ag85B peptide was the most immunodominant also in TB patients at T0 and at T4, as estimated by enumerating the frequencies of tetramer-specific CD8 T-cells; however significant differences in frequencies of epitope-specific CD8 T-cells were observed in TB patients before and after chemotherapy. In three instances (Esat-6, Rv1490 and 16 kDa antigens), mean frequencies of epitope-specific CD8 T-cells significantly increased after therapy: the mean frequency of Esat-6-specific CD8 T-cells was 0.39% in patients at T0 and 0.55% in patients at T4 (p<0.02), the mean frequency of Rv1490-specific CD8 T-cells was 0.35% at T0 and raised to 0.41% at T4 (p<0.05), the mean frequency of 16 kDa-specific CD8 T-cells was 0.24% at T0 and 0.38% at T4 (p<0.05) and the mean frequency Ag85B-specific CD8 T cells was 0.65% at T0 and 0.78% at T4. However, the frequencies of CD8 T-cells specific for the two other studied epitopes remained virtually unchanged before and four months after therapy: in fact, the mean frequency of Rv1614-specific CD8 T-cells was 0.38% at T0 and 0.41% at T4, and finally, the mean frequency of Hsp65-specific CD8 T-cells was 0.52% at T0 and 0.55% at T4.

**Figure 1:** Comparison of the frequencies of tetramer^+^ CD8 T-cells in peripheral blood from LTBI subjects and TB patients with active disease before therapy (T0) and after four months of therapy (T4). (A) In each group tested, LTBI subjects, TB patients at T0 and TB patients at T4, the median proportion of tetramer^+^ CD8 T-cells was estimated as 100% and the relative percentages of individual tetramer^+^ CD8 T-cells calculated accordingly. (B) Dot plot analysis of tetramer^+^ CD8^+^ T-cell populations of one representative LTBI subject, one TB patient at T0 and one TB patient at T4.

Figure 1B shows FACS analysis of the tetramer^+^ CD8^+^ T-cells of one representative LTBI subject, one TB patient at T0 and one TB patient at T4.

Altogether, these results indicate that (a) the frequencies of Mtb epitope-specific CD8 T-cells during active pulmonary TB disease in adults are lower than in LTBI individuals, but that they increase after anti-mycobacterial therapy; (b) that between 50 and 100% of epitopes selected are recognized by individuals with latent or active Mtb infection, including two new epitopes (Rv1490 and Rv1614) and (c), that there appears to be an immunodominance hierarchy in the recognition of different epitopes of Mtb in individuals with LTBI, as well as in patients with active TB before and after therapy.

### Phenotypic analysis of tetramer-specific CD8 T-cells

CD8 T-cells can be divided into at least four different populations of naive, central memory, effector memory and terminally-differentiated effector memory T-cells, based on the expression of surface markers associated with their maturation [16]. We have compared the phenotype of circulating tetramer-specific CD8 T-cell subsets in HLA-A*0201 TB patients at T0 and T4 and in individuals with LTBI. Representative data are shown in Figure 2A and cumulative data are shown in Figure 2B.

**Figure 2:** Phenotypic analysis of tetramer^+^ Mtb-specific CD8 T-cells. Peripheral blood mononuclear cells (PBMC) were stained with individual tetramers, and anti-CD8, -CD45RA and -CCR7 mAbs to separate functionally distinct subpopulations. After gating on tetramers^+^ CD8^+^ cells, the percentage of cells expressing CD45RA and CCR7 was determined. (A) Representative phenotyping data for one subject with LTBI (LTBI), one TB patient before (T0) and one TB patient 4 months after therapy (T4). Numbers in the corners indicate the percentage of positive cells in each quadrant. (B) Summary cumulative data of the phenotype of tetramer^+^ Mtb-specific CD8 T-cells. Data are presented with box plot reporting the median values and the interquartile range. Black columns = LTBI; grey columns = T0; white columns = T4.

The mean frequencies of tetramer-specific CD8 T-cells with a CCR7^+^ CD45RA^+^ naive phenotype were found to be comparable in TB patients and in subjects with LTBI. However, in the latter we found that approximately 60% of CD8 T-cells expressed CD45RA but not CCR7, indicating a terminally-differentiated phenotype; this was irrespective on their antigen specificity. In LTBI subjects, about 5% of the specific CD8 T-cells had an effector memory-like phenotype (CD45RA^−^ CCR7^−^), while less than 5% had a central memory-like phenotype (CD45RA^−^ CCR7^+^).

In TB patients, although cells expressing a terminally-differentiated CD45RA^+^ CCR7^−^ phenotype still comprised the predominant subset among specific CD8 T-cells, their mean percentage was lower than in subjects with LTBI (35% *versus* 60%) and remained virtually unchanged before and four months after therapy (35% *versus* 42%). However, although lower percentages of CD45RA^+^ CCR7^−^ cells was detectable within all studied tetramer^+^ CD8 T-cells, none of the differences between LTBI subjects and TB patients before or after therapy attained statistical significance. Conversely, tetramer-specific CD8 T-cells from TB patients contained higher proportions of cells with an effector memory-like (15% in TB patients *versus* 5% in LTBI subjects) and a central memory-like (10% in TB patients *versus* 3% in LTBI subjects) phenotype; however, also the frequencies of these two memory subsets did not change significantly before and after therapy. Thus, the data here reported also point to qualitative differences between TB patients and LTBI subjects in their antigen-specific CD8 T-cell compartment and suggest that the pool of terminally-differentiated CD45RA^+^ CCR7^−^ epitope-specific CD8 T cells is reduced in TB patients.

### Analysis of cytokine production by peptide-specific CD8 T-cells at the single cell level

IFN-γ and IL-2 have been shown to be the most relevant cytokines to define functional populations of antigen-specific CD4 and CD8 T-cells [16]–[18]. With regard to CD8 T-cells, two cell populations can be defined on the basis of the ability to secrete IL-2 and IFN-γ: CD8 T-cells secreting simultaneously IL-2 and IFN-γ (dual IL-2^+^/IFN-γ^+^), and CD8 T-cells secreting only IFN-γ (single IFN-γ). To assess these two profiles, we stimulated PBMC of HLA-A*0201 LTBI subjects and TB patients with the same individual peptides as those present in tetramers used in this study and determined the proportion of tetramer specific CD8 T-cells that produced IFN-γ and/or IL-2 by intracellular FACS analysis, after short-term stimulation with peptides. Representative data are shown in Figure 3A and cumulative data are shown in Figure 3B.

**Figure 3:** Polyfunctional cytokine production analysis of tetramer^+^ Mtb-specific CD8 T-cells. Peripheral blood mononuclear cells (PBMC) were stimulated with the same individual peptides as those present in tetramers and were stained with mAbs to CD8, IFN-γ and IL-2, or with isotype-control mAbs. After gating on CD8^+^ cells, the percentage of cells expressing IFN-γ and IL-2 was determined. (A) Representative intracellular cytokine staining data in one subject with LTBI, one TB patient before therapy and one PPD^−^ healthy donor. Numbers in the corners indicate the percentage of CD8^+^ cytokine-positive cells in each quadrant. (B) Summary cumulative data of the IFN-γ and IL-2 secretion capability of tetramer^+^ Mtb-specific CD8 T-cells in LTBI subjects (white bars) and TB patients with active disease before therapy (black bars). The data are expressed as the percentage of CD8^+^ T-cells that are IFN-γ^+^/IL-2^−^ or IFN-γ^+^/IL-2^+^. The values reported are the mean percentage of the different subset analysed for each group tested ± standard deviations (SD). *p<0.001 and **p<0.01 when compared to values in LTBI subjects.

Irrespective of the peptide, in subjects with LTBI 35%–45% of CD8 T-cells secreted both IL-2 and IFN-γ. The remainder of CD8 T-cells (55% to 65%) secreted only IFN-γ. In contrast, TB patients had a lower frequency of single IFN-γ-secreting cells against all tested peptides, but attained statistical significance only for Hsp65 peptide-specific CD8 T-cells. However, the most impressive finding was the consistent reduction of dual IL-2^+^/IFN-γ^+^ cytokine-secreting CD8 T-cells in TB patients, highly suggestive of a more restricted functional profile of Mtb-specific CD8 T-cells during active disease. Because of limited blood sample volume, it was possible to do intracellular cytokine staining after therapy only in five out of the patients at the first study time point. The results obtained showed, that four months after therapy all these five patients had still a dominance of IFN-γ-only secreting cells for all peptides tested except for the 16 kDa peptide. However, the limited number of patients after therapy did not allow statistical analysis of data.

These results indicate for the first time that the percentage of double IFNγ^+^/IL-2^+^ producing CD8 T-cells is significantly higher in LTBI subjects than in TB patients before therapy, suggesting a protective role of the two cytokines jointly in association with antigen specific CD8^+^ T-cell responses towards Mtb in latently infected healthy subjects. Figure 4 shows peptide-specific CD8 T-cell producing single IFN-γ^+^ or double IFN-γ^+^/IL2^+^: each portions of a pie chart indicates the mean percentage of peptides-specific T cells that responded with one or two functions.

**Figure 4:** Peptides-specific CD8 T cell responses in LTBI subjects, in TB patients at T0 and T4. Peptides-specific CD8 T cell responses are shown as a pie chart. Each portion of a pie chart indicates the percentage of peptides-specific T cells that responded with one or two functions, i.e. producing IFN-γ alone or the combination of IFN-γ and IL-2 (see legend).

## Discussion

CD8 T-cells play a critical role in chronic viral infection, but during recent years their role has gained increasing attention also in Mtb infection. In the present study, we investigated the *ex-vivo* frequencies, multifunctional cytokine production and memory phenotype of circulating CD8 T-cells specific for different peptide-nonamers of Mtb proteins in adult HLA-A*0201 subjects with LTBI and in TB patients before (T0) and after four months of anti-mycobacterial therapy (T4).

The *ex-vivo* frequencies of circulating tetramer specific CD8 T-cells in TB patients before therapy was lower than in LTBI subjects, but increased at four months after therapy to comparable percentages detected in subjects with LTBI; this pattern was consistently found for all tested tetramers. Thus, the frequency of circulating Mtb-specific CD8 T-cells is halved during active TB, compared to LTBI individuals. The reason of the reduced antigen-specific CD8 T-cell frequencies in TB patients at the beginning of therapy and their recovery after four months is not known, but the simplest explanation is that in TB patients large numbers of CD8 T-cells are sequestered at the site of disease and repopulate the peripheral blood compartment after successful anti-mycobacterial therapy. The phenomenon of sequestration of antigen-specific cells has been widely observed in TB for both CD4 and CD8 T-cells [14], [19], [20].

The data here reported also point to qualitative differences between TB patients and LTBI subjects in their antigen-specific CD8 T-cell compartment: while approximately 60% of antigen-specific CD8 T-cells in LTBI expressed a terminally-differentiated phenotype (CD45RA^+^CCR7^−^), in TB patients this was only 35% of antigen-specific CD8 T-cells. Conversely, TB patients had higher proportions of cells with an effector memory-like and a central memory-like phenotype. Interestingly, the phenotype of the CD8 T-cell population did not change significantly four months after therapy. These findings are somewhat surprising on the basis of our previous study of CD8 T-cell phenotype in children with TB, where the antigen-specific CD8 T-cell distribution pattern consistently changed four months after therapy, with a significant recovery of terminally differentiated effector memory T-cells and decreased frequencies of central memory T-cells [14]. Another study reported expansion of effector-memory CD8 T-cells in children with TB [15], which express a CD28 and CD27 double negative phenotype. However, care should be taken in correlating the phenotype with the functional properties. For instance, CD45RA^hi^ CD8 T-cells may accumulate during chronic viral infections in elderly individuals representing a pool of apoptosis-resistant memory cells that retain replicative potential [21].

The reason for the reduction of antigen-specific CD8 T-cells during active TB is unknown. As discussed above, one explanation we favour is that these cells are sequestered at sites of infection. Accordingly, a significantly high percentage of Mtb Ag85A epitope-specific CD8 T-cells was previously reported in the cerebrospinal fluid (CSF) of a child with TB meningitis [14].

Alternatively, it is possible that the low frequency of specific CD8 T-cells in active TB could be the consequence of sustained *in vivo* mycobacterial stimulation, which causes their apoptosis. For example, high levels of bacteria (such as occurs in TB patients due to the inability to contain and prevent their spread) could result in chronic stimulation of CD8 T-cells and induce their apoptosis.

A final aim of our study was to assess the capability of Mtb-specific CD8 T-cells to coproduce IFN-γ and IL-2, which is thought to be an indication of their multi-functionality and which has been associated with protective immunity [22]. Our results show that while in subjects with LTBI there was a high percentage of IL-2^+^/IFN-γ^+^ and IL-2^−^/IFN-γ^+^ peptide-specific CD8 T-cells, the IL-2^+^/IFN-γ^+^ population was consistently reduced in TB patients, highly suggestive of a restricted functional profile of Mtb-specific CD8 T-cells during active disease. While to our knowledge there has been no study comparing the cytokine response of CD8 T-cells at a single cell level in LTBI subjects and patients with active TB, a recent study on the CD4 T-cell response to Esat-6 and CFP-10 reported that there was a shift in the IFN-γ and IL-2 cytokine profile, notably from a dominance of IFN-γ-only T-cells in active tuberculosis to a dominance of IFN-γ/IL-2-double secreting T-cells [18]. These results, together with those reported in this paper, suggest distinct T-cell functional signatures between subjects which control Mtb infection (LTBI individuals) and those who do not (active TB disease). Accordingly, studies on CD8 T-cell responses in chronic infections such as HIV, CMV, EBV and HCV [23], [24] have highlighted signatures of protective antiviral immunity: poly-functional (i.e. IL-2 and IFN-γ secretion) and not mono-functional (i.e. IFN-γ only secreting) CD4 and CD8 T-cell responses represent correlates of protective antiviral immunity in chronic viral infections. Furthermore, the levels of antigen load modulate the phenotypic and functional patterns of the T-cell response within the same virus infection. Accordingly, Lalvani and colleagues demonstrated that functional CD4 T-cell heterogeneity is also associated with changes in Mtb antigen load: in active disease, in which antigen load if high, IFN-γ is secreted from two functional subsets, namely IFN-γ-only and IFN-γ/IL-2 dual secreting T-cells, whereas after therapy when antigen load is low, IFN-γ is predominantly secreted from IFN-γ/IL-2 dual secreting CD4 T-cells [18].

Although more extensive phenotyping of Mtb-specific IFN-γ- and IL-2-secreting T-cells is beyond the scope of this study, previous studies have identified a relationship between the function and phenotype of memory CD4 T-cells and proposed that the IL-2-only secreting cells are typical of central memory T-cells that persist after antigen clearance while the IFN-γ/IL-2- and IFN-γ-only secreting T-cells are typical of effector memory T-cells [20], [22]. Accordingly, a recent paper reported that in children vaccinated with BCG, specific CD8 T-cells identified by intracellular IFN-γ secretion, displayed a predominant CD45RA^−^CCR7^−^ effector memory phenotype, while a central memory population (CD45RA^−^CCR7^+^) was the second most common [25].

Phenotypic and functional signatures of CD8 T-cells could be used as an immunological marker of mycobacterial load, to monitor the response to treatment, to evaluate new therapies for active tuberculosis and the efficacy of new vaccines in clinical trials where new biomarkers are needed. Moreover, phenotypic and functional signatures of CD8 T-cells could also be used to monitor individuals latently infected with Mtb at a high risk of progression to active tuberculosis, such as those with HIV coinfection or on anti-TNF therapy.

## Materials and Methods

### Human subject

Peripheral blood was obtained from 13 HLA-A*0201 positive adults with TB disease (7 men, 6 women, age range 50–58 years) from the Dipartimento di Medicina Clinica e delle Patologie Emergenti, University Hospital, Palermo, and Monaldi Hospital, Naples, Italy, and 9 HLA-A*0201 LTBI subjects (5 men, 4 women, age range 30–45 years) and 5 tuberculin (PPD)^−^ negative healthy subjects (3 men, 2 women, age range 35–55 years). TB patients had clinical and radiological findings consistent with active pulmonary TB [26]. Diagnosis was confirmed by bacteriological isolation of Mtb in 12 patients and 1 further patient was classified as having highly probable pulmonary TB on the basis of clinical and radiological features highly suggestive of TB that were unlikely to be caused by another disease and a decision was made by the attending physician to initiate anti-tuberculosis chemotherapy, which resulted in an appropriate response to therapy. All patients were treated in accordance with italian guidelines and received therapy for 6 months. Treatment was successful in all participants as evidenced by no clinical or radiographic evidence of current disease, the completion of anti-tuberculosis chemotherapy and sterile mycobacterial cultures. Peripheral blood was collected before (T0) and 4 months after chemotherapy (T4). The follow-up time point of four months after starting therapy following was chosen on the basis of previous studies by our and other groups [19], [27]–[29] which have demonstrated change in many different immune responses in TB patients at this time point after therapy, including the CD8 T cell phenotype in childhood TB [14]. None of the TB patients had been vaccinated during infancy with BCG, or had evidence of human immunodeficiency virus (HIV) infection, or was being treated with steroid or other immunosuppressive or anti-tubercular drugs at the time of their first sampling. Tuberculin (purified protein derivative, PPD) skin tests were considered positive when the induration diameter was larger than 5 mm at 72 hrs since injection of 1 U of PPD (Statens Seruminstitut, Copenaghen, Denmark). The study was approved by the Ethical Committee of the Dipartimento di Medicina Clinica e delle Patologie Emergenti, University Hospital, Palermo, and Monaldi Hospital, Naples, Italy where the patients were recruited. Informed consent was written by all participants.

For the identification of LTBI subjects, in the absence of a gold standard, the most widely used diagnostic test remains the tuberculin skin test, based on the delayed-type hypersensitivity reaction that develops in Mtb infected individuals upon intradermal injection of PPD. However, this test suffers from many limitations, including false-negative results, especially in some high-risk groups, and false-positive results in BCG-vaccinated individuals or in subjects exposed to non-tuberculous mycobacteria [30]. Moreover, *in vitro* release of IFN-γ by T lymphocytes upon stimulation with the Mtb-specific antigens Esat-6 and CFP-10 (the T-SPOT.TB test-Oxford Immunotec, Oxford, United Kingdom and the QuantiFERON-TB Gold test-QFT-G, Cellestis, Victoria, Australia), was performed for all patients, for all LTBI subjects that resulted positive, and for PPD^−^ healthy donors included in the present study [31], [32].

Individuals with LTBI were defined as healthy people with a positive tuberculin skin test and no symptoms and signs of active TB. All of the LTBI subjects were health care workers, and thus very likely to be close contacts of TB index cases. Moreover, all the LTBI subjects included in this groups have not been vaccinated with BCG.

All the subjects were HLA typed serologically. The HLA subtype, A*0201, was confirmed by PCR amplification technique using sequence-specific oligonucleotide primers.

### HLA-A*0201 and β2-microglobulin

Recombinant HLA-A*0201 was over expressed in *E. coli*, purified as described [33] and dissolved in 8M urea. The integrity of the protein was confirmed by TOF-MALDI mass spectrometry using insulin as an internal reference. Human β2-micro-globulin was purchased from Sigma (St. Louis, MO) and dissolved in H_2_O. Heavy chain (50 µM) stock solutions were stored at −20°C until use.

### Synthetic peptides

A total of 6 nonamer peptides derived from the sequence of the proteins of Mtb and containing HLA-A*0201-binding motifs [34] were prepared using solid-phase/Fmoc chemistry, as described in detail elsewhere [19], [35], [36]. The peptides were of 90% purity, and their homogeneity was confirmed by analytical reverse-phase high-performance liquid chromatography, mass spectroscopy, and amino acid composition analysis. The sequences of the peptides were: Ag85B p5–13 (GLPVEYLQV), Esat-6 p82–90 (AMASTEGNV), Hsp65 p362–370 (KLQERLAKL), 16 kDa p120–128 (GILTVSVAV), Rv1490 p325–333 (FLLGLLFFV) and Rv1614 p197–205 (FLYELIWNV). Whereas the former 4 peptides have been identified previously, the latter two are newly identified in this study as candidate epitopes, based upon whole Mtb genome screening for 9-mer peptides sequences with the high and intermediate predicted HLA-A*0201 binding affinity as indicated in Table 1.

The two peptides derived from Rv1490 and Rv1614 were identified after a full genome-wide screening with the HLA_BIND algorithm. The two selected peptides had the highest predicted score for binding to HLA-A*0201, and there are reported strong associations between peptide binding HLA-A*0201 affinity and epitope recognition for CD8 T-cells in tuberculosis [37]. The *in silico* approach matched the strategy previously used to identify CD8 T-cell epitopes across the entire Mtb genome [17], [38].

Candidate HLA-A*0201 binding peptides in Hsp65 were selected using the MOTIFS software described previously [39]. Positive scores were given for each potential anchor residue found in the peptide, and negative scores were given to inhibitory residues. The overall peptide score was the sum of the scores for individual anchor and inhibitor residues.

### HLA-A*0201-peptide binding assay

HLA-A*0201 was titered in the presence of 100 fmol standard peptide to determine the HLA concentration necessary to bind 20–50% of the total fluorescent signal [35]. All subsequent inhibition assays were then performed at this concentration. HLA-A*0201 was incubated in 96-well plates (polypropylene, serocluster, Costar) at RT (pH 7) for 24 h with 0.5 µl β2M (15 pmol) and 1 µl (100 fmol) fluorescent labelled peptide in 92.5 µl assay buffer (100 mM Na-phosphate, 75 mM NaCl, 1 mM CHAPS), 2 µl protease inhibitor mixture (1 µM chymostatin, 5 µM leupeptin, 10 µM pepstatin A, 1 mM EDTA, 200 µM pefabloc) and 2 µl of the peptides of which HLA-binding capacity was to be determined. As a standard peptide we used FLPSDC(Fl)FPSV. The HLA-peptide complexes were separated from free peptide by gel filtration on a Synchropak GPC 100 column (250 mm×4.6 mm; Synchrom, Inc., Lafayette, Indiana). Fluorescent emission was measured at 528 nm on a Jasco FP-920 fluorescence detector (B&L Systems, Maarssen, The Netherlands). As HPLC running buffer, assay buffer containing 5% CH_3_CN was used. The percentage of labelled peptide bound was calculated as the amount of fluorescence bound to MHC divided by total fluorescence. The concentration of peptide inhibitor yielding 50% inhibition (IC50) was deduced from the dose-response curve. Each peptide was tested in at least two separate experiments. Data are expressed as relative (rel) IC50, compared to the IC50 of the standard peptide HBV core p47–56, which was considered as 1. Binding affinities of peptides to the HLA-A*0201 molecule were defined as high (IC50<1 µM), intermediate (IC50 1–10 µM) and low (IC50>10 µM). Note that, although the binding affinity of the Ag85 peptide is intermediate, it has been shown that is able to induce potent CD8 CTL activity [35].

### Generation of HLA-A*0201-Peptide Tetramers

Tetrameric HLA-A2-peptide complexes were prepared as follows: recombinant HLA-A*0201 and human β2-microglobulin, produced in *Escherichia coli*, were solubilized in urea and injected together with each synthetic peptide into a refolding buffer consisting of 100 mM Tris (pH 8.0), 400 mM arginine, 2 mM EDTA, 5 mM reduced glutathione, and 0.5 mM oxidized glutathione. Refolded complexes were purified by anion exchange chromatography using DE52 resin (Whatman) followed by gel filtration on a Superdex 75 column (Amersham Pharmacia Biotech). The refolded HLA-A*0201-peptide complexes were biotinylated by incubation for 16 hrs at 30°C with BirA enzyme (Avidity, Denver). Tetrameric HLA-peptide complexes were produced by the stepwise addition of extravidin-conjugated phycoerythrin (PE) (Sigma) to achieve a 1∶4 molar ratio (extravidin-PE/biotinylated HLA class I). The PE-labelled HLA-A*0201 tetramer complexed with the HIV-1 gag peptide p76–84 (SLYNTVATL was obtained from Proimmune Ltd. (Oxford, UK) and used as a negative control of tetramer staining.

### Tetramer staining and immunophenotyping

PE-labelled HLA-A*0201 tetramer complexes loaded with the Mtb peptides Ag85B p5–13 (GLPVEYLQV), Esat-6 p82–90 (AMASTEGNV), Hsp65 p362–370 (KLQERLAKL), 16 kDa p120–128 (GILTVSVAV), Rv1490 p325–333 (FLLGLLFFV) and Rv1614 p197–205 (FLYELIWNV) were used throughout. Tetramer staining was carried out as described in detail previously: peripheral blood mononuclear cells (PBMC) were isolated from heparinized blood samples by Ficoll-Hypaque (Sigma) density centrifugation. PBMC were incubated in U-bottom 96-well plates, washed twice in phosphate buffered saline (PBS, Euroclone, Milan, Italy) containing 1% fetal calf serum (FCS, Sigma) and stained for 30 min at 4°C with PE-labelled tetramers (3 µl), washed and subsequently stained with FITC-labelled anti-CD8 mAb (clone HIT8a, BD Biosciences, San Josè, CA) and analyzed by flow cytometry on a FACS Calibur analyzer with the use of the CellQuest software (BD Biosciences). Viable lymphocytes were gated by forward and side scatter and the analysis was performed on 100.000 acquired events for each sample.

To assess the phenotype of tetramer^+^ T-cells, cells were stained with FITC-labelled anti-CD8 mAb, APC-labelled anti-CCR7 (clone 3D12) mAb and PE-Cy5-labelled anti-CD45RA mAb (clone HI100) all from BD Biosciences in incubation buffer (PBS-1% FCS-0,1% Na azide) for 30 min at 4°C. Cells were then washed twice in PBS 1% FCS and analyzed by flow cytometry as previously described. Analysis was performed on 100.000 acquired events for each sample.

### Intracellular cytokine staining

PBMC (10^6^/ml) were stimulated with peptides (1 µg/ml, final concentration), in the presence of monensin for 6 hrs at 37°C in 5% CO_2_. The cells were harvested, washed and stained with APC-conjugated anti-CD8 mAb (BD) in incubation buffer (PBS-1% FCS-0.1% Na azide) for 30 min at 4°C. The cells were washed twice in PBS-1% FCS and fixed with PBS-4% paraformaldehyde overnight at 4°C. Fixation was followed by permeabilization with PBS–1% FCS–0.3% saponin–0.1% Na azide for 15 min at 4°C. Staining of intracellular cytokines was performed by incubation of fixed permeabilized cells with PE-labelled anti-IFN-γ (clone B27) and FITC-labelled IL-2 antibody (clone MQ1-17H12) or an isotype-matched control mAb. All mAbs were from BD Biosciences. Cells were acquired and analysed by FACS as described above.

### Statistical considerations

Negative control (background) values for cytokine staining were not subtracted from peptide-induced responses. For phenotype distribution analysis we used a cut off of a minimum number of 50 events, with a mean of 250 events for all tetramers tested and for each group of individuals tested.

Nonparametric Mann-Whitney U test was used to determine statistical differences in the distribution of the results. Values of *p*<0.05 were considered significant. Data were analyzed using statistical software SYSTAT 11 (Systat Software).
